This article has been retracted.

# Novel splicing variant c. 208+2T>C in *BBS5* segregates with Bardet–Biedl syndrome in an Iranian family by targeted exome sequencing

**DOI:** 10.1042/BSR20181544

**Published:** 2019-03-29

**Authors:** Saber Imani, Jingliang Cheng, Jiewen Fu, Abdolkarim Mobasher-Jannat, Chunli Wei, Saman Mohazzab-Torabi, Khosrow Jadidi, Mohammad Hossein Khosravi, Marzieh Dehghan Shasaltaneh, Lisha Yang, Md. Asaduzzaman Khan, Junjiang Fu

**Affiliations:** 1 Key Laboratory of Epigenetics and Oncology, Research Center for Preclinical Medicine, Southwest Medical University, Luzhou, Sichuan, China; 2 Institute of Medical Technology, Xiangtan Medicine and Health Vocational College, Xiangtan, Hunan, China; 3 Student Research Committee, Baqiyatallah University of Medical Sciences, Tehran, Iran; 4 State Key Laboratory of Quality Research in Chinese Medicine, Macau Institute for Applied Research in Medicine and Health, Macau University of Science and Technology, Macau (SAR), China; 5 Noor Ophthalmology Research Center, Noor Eye Hospital, Tehran, Iran; 6 Department of Ophthalmology, Bina Eye Hospital Research Center, Tehran, Iran; 7 Department of Biology, Faculty of Science, University of Zanjan, Zanjan, Iran

**Keywords:** Bardet-Biedl syndrome, BBS5 gene, Splicing variant, Targeted exome sequencing

## Abstract

Bardet–Biedl syndrome (BBS) is a rare genetically heterogeneous ciliopathy which accompanies retinitis pigmentosa (RP). However, the BBS5 mutation remains unclear in Iranians with BBS. The purpose of study is to evaluate genetic analyses of a BBS Iranian family using targetted exome sequencing (TES). A male 11-year-old proband and three related family members were recruited. Biochemical tests, electrocardiography and visual acuity testing, such as funduscopic, fundus photography (FP), optical coherence tomography (OCT), and standard electroretinography, were conducted. Molecular analysis and high-throughput DNA sequence analysis were performed. The proband was diagnosed with possible BBS based on the presence of three primary features and two secondary features. The TES analysis of the proband with BBS resulted in the identification of a novel, homozygous splicing variant c. 208+2T>C of the *BBS5* gene (NM_152384.2) in this Iranian BBS family. This variant was confirmed and was completely co-segregated with the disease in this family by Sanger sequencing. Thus, we report a novel, homozygous splicing site variant c.208+2T>C in the *BBS5* gene for the first time in the Iranian family.

## Introduction

Mutations in approximately 250 genes have been identified to cause inherited retinal dystrophies, leading to clinically and genetically heterogeneous group of disorders [1]. Retinitis pigmentosa (RP) (OMIM: 268000) accounts for approximately one-half of the cases. According to current research, approximately 3100 reported mutations in more than 50 genes cause non-syndromic RP [2,3] and syndromic forms of RP, including Usher syndrome (USH) (OMIM: 276900) and Bardet–Biedl syndrome (BBS; OMIM: 209900). Mutations in 12 genes are associated with USH and 21 genes cause BBS; together, these two diseases consist of 1200 pathogenic mutations [4].

BBS is a very rare (1:13500–1:160000) autosomal recessive pleiotropic disorder. It is both genetically and clinically heterogeneous [4,5]. This multi-systemic developmental disorder is primarily characterized by rod-cone dystrophy (frequency: 93%), polydactyly (frequency: 63–81%), obesity (frequency: 72–92%), genital anomalies (frequency: 59–98%), renal anomalies (frequency: 53%), cognitive impairment, and learning difficulties (frequency: 61%) [6,7]. In addition, secondary characteristics include liver abnormality, diabetes mellitus, slow growth, psychomotor delay, speech disorder, developmental delay, strabismus, dental disorders, hearing loss and cardiac malformations. A BBS diagnosis can be made with the presence of at least four primary features, or three primary plus two secondary features.

*BBS-5* gene (*BBS5*; NM_129880, OMIM: 603650), which encodes protein BBS5, is directly linked to BBS [8,9]. The BBS5 is associated with ciliary trafficking, ciliogenesis, and regulation of sonic hedgehog signal transduction, and is one of the seven essential proteins to form BBSome [10,11]. BBS5 contains two pleckstrin homology-like domains and binds to phosphoinositides, which is critical for ciliogenesis [12]. The *bbs5* gene knockout in mice lead to abnormalities like obesity, impaired glucose homeostasis, and abnormal retinal morphology [13]. BBS5 is a minor contributor to BBS as only 2% of families from various ethnic backgrounds harbored *BBS5* variants [9]. Up till now, different types of variants in the *BBS5*, such as missense, nonsense, deletions, and insertions, have been reported that are directly or indirectly involved in syndromic retinal dystrophy disease such as RP (OMIM: 268000) and cone-rod dystrophy (CRD, OMIM: 120970), and other diseases such as polydactyly (OMIM: 603596) [11,14]. However, the implication of the *BBS5* gene variant in Iranian BBS patients is not well characterized.

The present study was aimed to provide genetic analyses of BBS using the next-generation sequencing (NGS) [15,16]. As shown in previous reports, NGS is a feasible and cost-effective technique with high coverage in a short reversal time and has been widely used in nationwide surveys of rare diseases [17,18]. Thus, here, we report the results of a novel homozygous variant in an Iranian clinically diagnosed family with multiple clinical feature of BBS phenotype.

## Materials and methods

### Ethics statement

The current study was approved by the ‘Ethics Review Board’ of the Southwest Medical University in China and local Ethics Committee guidelines of Ophthalmology Center, Bina Eye Hospital, Tehran, Iran, as well as followed the recommendations of the Helsinki declaration [19,20]. The family was informed in detail about the study and written consent forms were taken from all participants before the study.

### Family description, clinical assessment, and biochemical tests

An 11-year-old Iranian, the second of two children from a non-consanguineous marriage (proband, pedigree II:2 is depicted in Figure 1) and three related family members were recruited in the study (Figure 1). The patient has a poor vision since the age of 4 and it worsened with time since then. He underwent through assessment and the BBS diagnosis was made based on previously described criteria [2].

**Figure 1:** The pedigree in an Iranian family with BBS Affected individuals and carriers are shown as filled and as semi-filled symbols, respectively. The patient above the arrow indicates the proband (II:2) with a variant of the *BBS5* gene: NM_152384.2:c.208+2T>C. ‘IRB’ means the molecular number in our collected sample database. ‘+’ indicates wild type allele, whereas ‘-’ indicates mutant type allele.

The biochemical tests, including hematologic tests (complete blood count), liver function tests (AST, ALT, alkaline phosphatase, PT/INR, and bilirubin), renal function tests (serum creatinine and urea), lipid panel tests (serum triglycerides, total cholesterol, HDL, and LDL), thyroid function tests (TSH, T3, T3RU, and T4), and gonadotropin levels, were performed. Brain was surveyed using magnetic resonance imaging (MRI) to determine probable malformations. Anatomical evaluation of internal organs was performed using abdominal and pelvic ultrasonography. The electrocardiography (ECG) and echocardiography were used for cardiac function evaluation.

Ocular abnormalities were diagnosed using refraction testing, visual acuity testing, Humphrey visual field testing, slit-lamp biomicroscopy, and fundoscopy. Moreover, fundus photography (FP, Spectralis; Heidelberg Engineering, Heidelberg, Germany), optical coherence tomography (OCT, Carl Zeiss, Germany), and standard electroretinography (ERG, RetiPort ERG System; Roland Consult, Wiesbaden, Germany) were done [19].

### DNA sampling and targetted-NGS analysis

The sequence analysis was performed using capture Agilent probes, as described in previously published studies [12,15,19,21]. A total of 200 μl of peripheral blood was taken from each patient or healthy individuals in EDTA vacutainers (Figure 1). Human genomic DNA was extracted from leukocytes using standard Qiagen DNA extraction kit according to the manufacturer’s specifications (Qiagen, Hilden, Germany) [19]. Illumina Exome Content Set (Catalog Illumina Inc., San Diego, CA, U.S.A.) was used for enriching coding regions and exon–intron boundaries of pathogenic mutations in BBS candidate genes (*BBS1, BBS2, ARL6, BBS4, BBS5, MKKS, BBS7, TTC8, BBS9, BBS10, TRIM32, BBS12, MKS1, CEP290, WDPCP, SDCCAG8*, and *NPHP1*) and RP genes; as well as sample preparation for the NGS reaction. The design of exome capture panels has been described in previous studies, according to the Illumina paired-end libraries [12]. Sequencing was performed on an Illumina HiSeq 2000 (Illumina, Inc., San Diego, CA), following the manufacturer’s protocols. Sequencing data were analyzed by capture Agilent probes and IGV (Integrative Genomics Viewer). Paired-end sequencing Illumina reads were aligned to the human hg19 reference genome. Variant frequency data were aligned to online control databases, such as Exome Aggregation Consortium (ExAC), 1000 Genome Project, CHARGE consortium, ANNOVAR [22], and ESP-6500 databases, to find the pathogenic mutations in BSS candidate genes with a minor allele frequency of more than 5%. Meanwhile BBS is rare Iranian macular degeneration (MD) or dystrophy disorder; variants and deep intrinsic exon–intron junctions were filtered out from following analysis by the criteria of a frequency higher than 1/400 and distance >10 bp, respectively.

### Variant verification and co-segregation analysis

Eventually, all the detected variants of NGS in the present study were confirmed by PCR amplification and conventional Sanger-based sequencing (3500DX ABI genetic analyzer, Foster City, U.S.A.) in the proband and his family members [23–25]. In this regard, the locus-specific primers for variant verification and co-segregation analysis were designed using online Primer3 program. All reactions were performed with two replicates per sample and a control for each test.

### *In silico* analysis of the BBS5 protein and its variant

*In silico* analysis of the BBS5 protein conserved domain and its variant 208+2T>C was performed on NCBI program. Identifying conserved domains were performed using the following website: https://www.ncbi.nlm.nih.gov/Structure/cdd/wrpsb.cgi?INPUT_TYPE = live&SEQUENCE = NP_689597.1.

## Results

### Distribution of family

The pedigree of this family with classical genetic BBS phenotype has been illustrated (Figure 1). Pedigree analysis in all affected members is consistent with the autosomal recessive mode of inheritance. The proband is an 11-year-old, overweight, Iranian male from the west part of Iran with a probed case of early clinical signs of progression in BSS at 4 years of age (Figure 1, II: 2). The parents belonged to a similar tribe with a same surname.

### Clinical findings

The demographic and clinical characteristics of BBS presented by patients have been shown in Table 1. The proband was obese (with a body mass index of 30.3) and he was attending school appropriate for his age but had speech delay and learning difficulty. During clinical examinations, the hypogenitalism was diagnosed in conjunction with biochemical hypogonadism. During dental examinations, dental anomalies including hypodontia and small roots were diagnosed. Other biochemical evaluations were in normal range and the brain MRI and abdominal and pelvic ultrasonography did not show any anatomical malformations. Cardiac evaluations were normal anatomically and functionally. Based on the presence of three primary features (obesity, hypogonadism, and retinal dystrophy) and two secondary features (speech delay and dental anomalies), thus the child was diagnosed with possible BBS (Table 1). The proband (pedigree II:2 is depicted in Figure 1) presented with a chief complaint of poor vision and night blindness since the age of 6, with best spectacle-corrected visual acuity of 4/10 in the right eye (OD) and 3/10 in the left eye (OS). The results of thyroid function tests (TSH, T3, T3RU, and T4) and gonadotropin levels were presented in Table 2, indicating that the testosterone level in the proband was decreased. The retinal phenotypes of all members of the family were compared with the ethically unaffected age-matched control in the Figure 2, respectively. Considerably, FP of the proband revealed bilateral optic nerve head pallor and retinal vascular attenuation (Figure 2B). Furthermore, FP image of anterior segments of the carrier case (pedigree I:1 is depicted in Figure 1) was remarkable only for pale optic disc, attenuated arterioles, trace bilateral subcapsular cataracts, and replacement of normal darkened presence (mainly in the right eye, Figure 2B). The comparison between two panels of the carrier and proband case of the BBS with normal control (Figure 2C) clearly showed the ‘salt and pepper’ pigment mottling pattern, central reddish orange hue, close mottling, severe retinal pigment epithelium (RPE) atrophic changes, and transparent in the macula (Figure 2).

**Figure 2:** Retinal phenotypes from patient, carrier and control Representative fundus photographs (FA) (**A**–**C**), OCT, and electroretinography (**D**–**F**). Representative fundus photographs (FA) from both eyes of the carrier for I:1 (A), proband for patient II:2 (B) in comparison with the fundus photographs of uninfected age-matched control (C). (D) Carrier for I:1. (E) Proband for patient II:2*.* (F) Unaffected age-matched normal control. Top panels indicate OCT and electroretinography features of inherited retinal dystrophies in the left eye. Bottom panels indicate OCT and electroretinography features of inherited retinal dystrophies in the right eye. OD in the left and OS in the right panels, respectively, have been presented.

**Table 1:** Clinical characteristics of BBS features presented by patients

Primary features	Pedigree II:2 (male)	Pedigree II:1 (female)
Retinal dystrophy	Yes	Yes
Age (years)	11	19
Body mass index	30.3	Not applicable
Obesity	Yes	Yes
Hypogonadism	Yes	Not applicable
Renal abnormality	No	Yes
Secondary features		
Speech disability	Yes	No
Strabismus, cataract, astigmatism	No	Posterior subcapsular cataract
Dental anomaly	Yes	No
Gastrointestinal problems	No	Digestion problem
Menstruation in females	-	Regular
Ophthalmic examinations		
Best corrected visual acuity	OD: -4.75-1.75 × 10 4/10	OD:- 2-3 × 160 CF 20-
	OS:-4.75-3.00 × 10 3/10	OS: -4 -2 × 10 CF 20-
Fundus appearance	Attenuated arterioles, Pale optic disc	Attenuated arterioles, Pale optic disc, Bone spicules, Macular atrophy
Initial symptom	Night blindness	Night blindness

**Table 2:** Biochemical and metabolic tests in the proband (Pedigree II:2)

Test in organs	Test type	Value	Normal range
Thyroid function tests	TSH	2 µlU/ml	(0.4–4.2 µlU/ml)
	T3	135 ng/dl	(80–210 ng/dl)
	Free T4	1.3 ng/dl	(0.8–1.5 ng/dl)
	Total T4	8.2 µg/dl	(5.6–11.7 µg/dl)
Gonadotropin profile tests	Testosterone	1.01 ng/ml	(1.50–9 ng/ml)

Macular OCT of the family has been shown in Figure 2D–F. Significant retinal thinning and RPE degeneration and the peripheral retina were observed in macula of both proband and his sister (Figure 2E, data not shown).

Loss of the outer retinal architecture, foveal atrophy of retina, and loss of normal foveal configuration of proband’s left eye are amongst extremely presented abnormalities. Considering both OD and OS image, cube average thickness of RPE lyres in the proband was significantly reduced compared with the normal case (158 compared with 273 μm). We found no significant change in cube average thickness of proband and carrier (158 compared with 230 μm). This figure proves the prospective disruption of the photoreceptor layer and choroidal that is increased by thinning in RPE. The proband’s sister (II:1 in Figure 1) was 19 years old, and had similar symptoms with proband. The parents did not show symptoms with proband.

### Targetted NGS analysis

To investigate the causative genes, targetted capture high-throughput genotyping was performed using an Illumina HiSeq 2000 sequencer. The proband was applied for target capture panel sequencing. This panel covers coding exons and flanking splicing junctions for 17 known BBS disease genes, including *BBS5*. The targetted regions with evenness scores more than 0.8 across of all samples were converged. Commonly, 96.0% of the targetted regions have a coverage >20× and 91.1% of the targetted regions have a coverage >40×. Ultimately, more than billion bases of sequence in 100-bp read length, 11400 Insertions/Deletions (INDELs), and 40000 single nucleotide polymorphisms (SNPs) were generated. After quality assessment, more than 97% of billions of bases were aligned with the human reference sequence, and amongst those, billion bases were covered with a ten-fold coverage target region. Variant annotation was performed using ANNOVAR [22] to annotate single nucleotide variants (SNVs) and INDELs, and RefSeq genes used as a reference to co-ordinate the mutations. Finally, sequence variants that were not annotated in any of the above public databases were prioritized for further characterizations. The targetted exome sequencing (TES) analysis of the proband (pedigree II:2 is depicted in Figure 1 and Supplementary Table S1), associated with BBS, resulted in the identification of a novel, splicing site variant 208+2T>C in *BBS5* (NM_152384.2) in this Iranian BBS family [26]. Variant location according to UCSC GRCh38/hg38 is in genomic Chr2: 169,487,136 (or UCSC hg19: Chr2: 170,343,646). Successfully, we identified the splicing variant c.208+2T>C in the intron 3 of *BBS5*. This variant may produce a novel splice site (a splice donor). This change has not been reported as an SNP.

### Verification and co-segregation analysis of *BBS5* gene

By high-quality NGS data identifying a variant in *BBS5*, c.208+2T>C, this splicing variant in *BBS5* gene was selected to verify and co-segregation analysis by Sanger DNA sequencing, according to the specific primers for the *BBS5* gene PCR amplification (sorted in Table 3). Sanger sequencing of the *BBS5* gene revealed a homozygous mutation of thymine nucleotide in intron 3 (c.208+2T>C) (Figure 3). This variant has been detected in heterozygous in proband’s parents (pedigree I: 1 and 2 is depicted in Figures 1 and 3A,B) and mutant homozygous type in proband’s sister and himself (pedigree II: 1 and 2 is depicted in Figures 1 and 3C,D). Thus proband (Figure 3D) and his sister (pedigree II: 1 Figures 1 and 3C) were homozygous for the variant of *BBS5*. Thus this variant, confirmed by Sanger sequencing, showed absolute co-segregation in pedigree association.

**Figure 3:** Sanger sequencing validation (**A**–**D**) Indicate the sequenced results in I:1, I:2 (mutant heterozygous type), II:1, II:2 (mutant homozygous type), respectively. The arrows indicate a novel splicing site variant at the nucleotide position c.208+2T>C in the *BBS5* gene. (**E**) The genomic region, including partial exon and intron sequences, with wild-type and mutant type of the *BBS5* gene. Arrow points the variant site. Abbreviations: Mut type seq, mutant type sequence; WT, wild-type.

**Table 3:** The sequences of PCR primers and PCR product sizes

Primer name	Left primer	Sequence (5′–3′)	Right primer	Sequence (5′–3′)	Size	°C
BBS5-BII2	BBS5-BII2L	ggccagaagttccatatcca	BBS5-BII2R	gcttcttccttctttgggatt	443	60
bbs5-RT	bbs5- RTL	gggagccccagactttttac	bbs5- RTR	catccgtgtggtcatcagag	547	60
RT-b-actin-m	RT-b-actin-mL	tgttaccaactgggacgaca	RT-b-actin-mR	tctcagctgtggtggtgaag	392	60

### *In silico* analysis of BBS5 protein and its variant

*In silico* analysis of conserved domain revealed that BBS5 is a BBL5 (BBS 5 protein) domain-containing protein (accession number: pfam07289) or belongs to BBL5 superfamily (Figure 4). BBS5 is part of the BBSome complex that may function as a coat complex required for sorting of specific membrane proteins to the primary cilia. BBS5 protein (NP_689597.1) has 341 amino acids in length (Figure 4). The splicing mutation might shift the reading frame and probably results in a truncated protein by skipping an exon, leading to loss of functional domains. The splicing site variant c.208+2T>C in the intron 3 resulted in amino acid changes after position 68 on BBS5 protein (Figure 4, arrow) and led to more than two-thirds of BBS5 C-terminus changes at least, or produced a truncated protein, likely a pathogenic variant. Comprehensively, BBS5 c.208+2T>C is mostly likely as a pathogenic variant, which leads to BBS in this Iranian family.

**Figure 4:** Human BBS5 protein conserved domain

## Discussion

In the current study we reported the genetic characterization of an Iranian family diagnosed with classic BBS. High-throughput NGS technique was used for the comprehensive assessment of coding regions and exon–intron boundaries of all identified BBS genes in this family. During the present study, we aimed to identify a probable novel disease-causing gene variant in the patient and his family members. According to targetted NGS results, a novel 208+2T>C homozygous splicing site mutation was identified in the *BBS5* gene. Up to now, 20 different mutations have been reported in the gene *BBS5* causing BBS including 12 missense/nonsense, 2 splicing and 6 deletion or insertion mutations. So, our reported mutation is the 21st mutation (third splicing mutation) of the gene *BBS5* leading to BBS.

The diagnosis of proband was based on three primary and two secondary criteria (RP, obesity, hypogonadism, speech disorder, and dental anomalies). In line with our projects upon the retinal dystrophy, complete clinical features analysis confirmed and revealed that ocular phenotype of this family correlated with mutations in distinct BBS genes, also most affected patients shared the classical features of BBS [12,15,27].

Genetically, BBS is one of the heterogeneous MD disorders [4,7]. More than 80% of clinically diagnosed BBS patients are supported by mutations in these selected BBS genes. Macular and retinal degeneration involvement appears to exacerbate with age in BBS and it is not frequently detected in patients under 4 years old.

Regarding this report and previous studies, essentially retinopathological investigations were driven by mutational data analysis from new molecular based diagnosis, such as NGS panel covering [23]. Furthermore, we proposed that macular progressive depigmentation with pigment clumping and atrophy is seen as a major complement in the proband, which was extremely apparent in the macula. These notwithstanding methods were able to screen and identify pathogenic mutations in inherited heterogeneous retinal disorders, such as RP, Stargardt disease (STGD)-like MD, leber congenital amaurosis (LCA), BBS, and USH [28,29]. It is clear that identification of new disease-causing variant has expanded the complexity of ciliopathies with respect to phenotypic variability, and thus pharmacologists have the chance to understand the distribution of mutations beyond the phenotyping of MD disease, primary fundamental locus, and expressivity [12,15,17,18]. To address this issue, by TGS-based models, we have succeeded in identifying a new *BBS5* disease-causing mutation in an Iranian BBS family (c. 208+2T>C), which broadened the mutant spectrum.

It has been widely accepted that different ethnic groups of the BBS patients have different frequencies of pathogenic variants in BBS genes. It has been recommended that molecular diagnosis could be recognized in more than 82% of BBS patients using a TES panel with known BBS genes [9]. Of note, *BBS4* and *BBS5* gene variants have been reported more frequently in Middle East countries [16]. Whereas in Indian population, variants were predominant in BBS10 and BBS3 genes; only one novel non-sense mutation c.425T>G; p(L142*) was obtained in BBS5 gene [30]. For the first time, the finding of *BBS5* c.208+2T>C variant, together with other reported variants in six other genes (*BBS3, BBS4, BBS6, BBS7, BBS9*, and *BBS12*) [31], proved the genetic heterogeneity of BBS in Iran, facilitating genetic counseling for this family.

The encoded protein of the *BBS5* gene, belonging to the BBSome complex, is essential for ciliogenesis. BBSome with mediated part of the Rab8 GDP/GTP exchange factor, facilitates the primary cilium and promotes extension of the ciliary membrane [10,32]. The BBSome complex is required for ciliary localization and assembly [9]. The recent report of Scheidecker et al. [33] functionally characterized the clinical features of the BBS patients with the mutations in the *BBS5* gene [33,34]. They found significant macular dystrophy in all patients, which typically presented with central hypofluorescence enclosed by an incessant hyperfluorescent ring on fundus autofluorescence imaging [33]. The splicing mutation might shift the reading frame and probably results in a truncated protein by skipping an exon, leading to loss of functional domains for forming the BBSome protein complex. Despite numerous genetic studies focussed on identifying of *BBS5* mutation (mainly deletion) in different MD degeneration, the molecular roles of these diseases are still unclear [34,35]. Furthermore, the full frequency spectrums of variations in this gene have not been reported in different ethnic groups of the BBS patients [9,33,34]. Imaginably as a result of the Iranian population’s complicated history, these findings could be a guide to reveal the phenotype–genotype correlation of BBS, besides primary features such as obesity and diabetes.

In conclusion, for the first time, we report a novel, homozygous splicing site variant c.208+2T>C in the *BBS5* gene in an Iranian family, which will help us understand the molecular mechanisms of BBS and facilitate gene diagnosis and genetic counseling.

## Supporting information

**Supplementary Table S1:** 

## Abbreviations

BBS: Bardet–Biedl syndrome
BBS5: BBS-5 gene
FP: fundus photography
INDEL: insertion/deletion
MD: macular degeneration
NGS: next-generation sequencing
OCT: optical coherence tomography
RP: retinitis pigmentosa
RPE: retinal pigment epithelium
SNP: single nucleotide polymorphism
TES: targetted exome sequencing
USH: Usher syndrome
